The article "Application of Ultrasound Virtual Reality in the Diagnosis and Treatment of Cardiovascular Diseases" was published in 2021. Journal: J Healthc Eng.

# Application of Ultrasound Virtual Reality in the Diagnosis and Treatment of Cardiovascular Diseases

**DOI:** 10.1155/2021/9999654

**Published:** 2021-08-17

**Authors:** Mingqiang Fan, Xiangxiang Yang, Tao Ding, Yu Cao, Qiaoke Si, Jing Bai, Yongchun Lin, Xinke Zhao

**Affiliations:** ^1^Cardiovascular Division, Pingliang People's Hospital, Pingliang 744000, Gansu, China; ^2^Cardiovascular Division, Affiliate Hospital of Gansu University of Traditional Chinese Medicine, Lanzhou 730020, Gansu, China

## Abstract

Cardiovascular disease is a common chronic disease in the medical field, which has a great impact on the health of Chinese residents (especially the elderly). At present, the effectiveness of the prevention and treatment of cardiovascular diseases in my country is not optimistic. Overall, the prevalence and mortality of CVD are still on the rise. The timely and effective detection and treatment of cardiovascular and cerebrovascular diseases are of great practical significance to improve the health of residents and to carry out prevention and treatment. This article aims to study the application of ultrasound-based virtual reality technology in the diagnosis and treatment of cardiovascular diseases to improve the efficiency and accuracy of the diagnosis of cardiovascular and cerebrovascular diseases by medical staff. The focus is on the application of feature attribute selection related algorithms and classification related algorithms in medical and health diagnosis systems, and a cardiovascular and cerebrovascular disease diagnosis system based on naive Bayes algorithm and improved genetic algorithm is designed and developed. The system builds a diagnostic model for cardiovascular and cerebrovascular diseases and diagnoses and displays the corresponding results based on the patient's examination data. This paper first puts forward the theoretical concepts of ultrasonic virtual reality technology, scientific computing visualization, genetic algorithm, naive Bayes algorithm, and surgery simulation system and describes them in detail. Then, we construct a three-dimensional ultrasonic virtual measurement system, from the collection and reconstruction of image data to the filtering and segmentation of image data, plus the application of three-dimensional visualization and virtual reality technology to construct a three-dimensional measurement system. The experimental results in this paper show that 10 isolated congenital heart disease models with atrial septal defect (ASD) established through the use of three-dimensional visualization and virtual reality technology measured the short diameter, long diameter, and area of the atrial septal defect in the left and right atria. Finally, a value of *L* less than 0.05 indicates that the statistics are meaningful, and a value of *r* generally greater than 0.9 indicates that the virtual measurement result is highly correlated with the real measurement result.

The article "Application of Ultrasound Virtual Reality in the Diagnosis and Treatment of Cardiovascular Diseases" was published in 2021. Journal: J Healthc Eng.

## 1. Introduction

Judging from the current situation, the number of cardiovascular diseases in China continues to increase, and this is one of the major causes of their deaths. From the comparative statistical analysis of the mortality rate of cardiovascular diseases and other diseases in China in recent years, it can be seen that, 100,000 as the base, compared with rural and urban, the CVD mortality ratio is 295.63 : 261.99, of which the heart disease mortality ratio is 143.72 : 136.21, the cerebral hemorrhage ratio is 74.51 : 52.25, and the cerebral infarction ratio is 45.30 : 41.99. This shows that cardiovascular disease is the number one killer of human health in the 21st century. Virtual reality (VR) is a technology that has developed rapidly in recent years. It has eliminated many industries through multiple advantages such as multimedia, multitasking, and effective interaction. Virtual reality technology can be roughly composed of desktop, immersive, distributed, and hybrid.

Cardiovascular function parameters are an important way to detect cardiovascular diseases. The detection is relatively accurate, but the risk is high, so it is only suitable for severely ill people and cannot be widely used in medical treatment. There are many methods to detect cardiovascular function clinically, including CT scan, electrocardiogram, echocardiography, and MRI. These methods can effectively detect cardiovascular function to effectively control cardiovascular disease, but these testing instruments are cumbersome and expensive, so they are not suitable for general household use.

Novo et al. introduced a web-based system called Hydra, which integrates a complete and detailed set of services and functions for clinical decision support to help and improve clinicians' diagnosis and risk assessment of cardiovascular patients over time. Work on treatment and monitoring: Hydra integrates many different services and also provides a set of reports derived from all the information collected by patients to support physicians' clinical decision-making. This platform improves the productivity and accuracy of patient data evaluation, but it is not practical in the real clinical medicine field [1]. This study by Pirani and Khiavi compares Iran's population percentages with those of the United States and Spain due to risk factors for cardiovascular disease. Finally, the research results show that, for people suffering from cardiovascular disease, blood pressure is the most important factor in cardiovascular disease that affects all risk factors. However, this study only discovered the biggest risk factor of cardiovascular disease through experiments and did not propose effective treatment measures [2]. Based on the knowledge that uric acid plays an important role in the pathogenesis of civilized diseases such as obesity, metabolic syndrome, and cardiovascular disease, ubica Cibiková and David Karásek believe that uric acid has become an independent risk factor for morbidity and mortality. It also leads to whether the relationship between uric acid and cardiovascular disease is direct (through the effects on endothelial dysfunction, oxidative stress and inflammation) or indirect (metabolic syndrome mediated by known cardiovascular disease risk factors, obesity, insulin resistance, and high blood pressure). However, based on current knowledge, it is impossible to recommend the treatment of hyperuricemia to reduce the risk of cardiovascular disease [3].

The article "Application of Ultrasound Virtual Reality in the Diagnosis and Treatment of Cardiovascular Diseases" was published in 2021. Journal: J Healthc Eng.

The innovation of this article is (1) using the visual advantages of virtual reality technology, combined with the special physiological mechanism of patients with cardiovascular diseases, to make up for the limitations of traditional treatment methods such as shortage of medical education resources, drug addiction, and safety issues, to provide patients with cardiovascular diseases and bring new, comprehensive, and efficient emerging treatment technologies. (2) Propose and design a cardiovascular and cerebrovascular disease diagnosis system based on the naive Bayes algorithm and improved genetic algorithm to assist in the diagnosis of cardiovascular and cerebrovascular diseases, avoiding medical staff due to their own subjective judgment and lack of clinical experience. Misdiagnosis, thereby, improves the efficiency and accuracy of disease diagnosis by medical staff and, at the same time, is of great significance to promoting the development of medical informatization.

## 2. Application Method of Ultrasound Virtual Reality Technology in the Diagnosis and Treatment of Cardiovascular Diseases

### 2.1. Ultrasonic Virtual Reality Technology

The clinical application value of two-dimensional ultrasound has been widely recognized. However, since the three-dimensional structure of the lesion cannot be visually represented by 2D cross-sectional images, 3D ultrasound imaging technology is required to solve these problems. 3D ultrasound imaging technology is developing rapidly, especially after the advent of real-time 3D ultrasound, and this 3D ultrasound technology has been successfully applied to heart disease and has produced excellent results. When this technology is combined with virtual reality technology, the virtual reality technology docks with auxiliary equipment such as control equipment, processes and calculates information through computer programs, and finally forms an interactive, simulating natural state and three-dimensional environment on the display terminal and making people Technology that creates a sense of immersion. The advantages of virtual reality technology, such as strong interest, high safety, and timely feedback, can break the limitations of traditional rehabilitation therapy and make up for its shortcomings. At the same time, virtual reality technology uses a computer simulation system to generate a simulation environment with its immersion and interactivity, and users can create and experience virtual worlds. It is an important cross-cutting technology for multisource information fusion [4, 5].

The article "Application of Ultrasound Virtual Reality in the Diagnosis and Treatment of Cardiovascular Diseases" was published in 2021. Journal: J Healthc Eng.

### 2.2. Visualization of Scientific Computing

The visualization of scientific computing is the use of computer graphics and image processing technology to convert a large amount of data generated by scientific engineering calculations into graphics and images for processing in an intuitive form. It refers to this theory, method, and technology. It belongs to an important research direction of graphics computers. In medicine, scientific visualization can use technologies such as ultrasound and ultrasound to capture 2D or 3D images, create 2D or 3D shapes, and display them on a computer. Based on this, computer simulations and surgical planning of orthopedic surgery and radiotherapy can be applied. Not only that, the real-time visualization of scientific computing also allows you to track the progress of functions on the screen during operation. This will greatly increase the success rate of surgery [6].

### 2.3. Genetic Algorithm

The American Professor Holland proposed this algorithm, Genetic Algorithm (GA), as early as 1975. This is a search algorithm that can be used to simulate the evolution of organisms in nature. Our country also published “Genetic Algorithm and Its Application” as early as 1996, and the professor of Tongji University put forward the idea of parallelization of genetic algorithm in 2002 [7, 8]. GA's ideas came from Darwin's biological evolution and Mendel's genetics. In essence, according to the evolutionary law of “survival of the fittest and survival of the fittest,” the excellent ones will get better and better, and the inferior ones will be eliminated gradually, and only the excellent ones will be left in the end. GA is widely used due to its simple, universal, and powerful other excellent features and has become one of the most important intelligent algorithms at the moment. At present, the main role of GA is feature selection and classification [9].

The article "Application of Ultrasound Virtual Reality in the Diagnosis and Treatment of Cardiovascular Diseases" was published in 2021. Journal: J Healthc Eng.

#### 2.3.1. Fitness Function

The fitness function is mainly used to evaluate the pros and cons of individuals, and the formula is shown in

(1) $$\begin{array}{c} f\left(a\right)=\frac{1}{1+e^{a}}. \end{array}$$

#### 2.3.2. Select Operation

The calculation formula for the expected value of the copy number of each individual is shown in (2), and the calculation result needs to be rounded:

(2) $$\begin{array}{c} S_{x}=S\frac{f_{x}}{\sum f_{x}}, \end{array}$$

*f*_*x*_ represents the fitness value of the *x*th individual, and *S*_*x*_ represents the sum of the population fitness.

### 2.4. Naive Bayes Algorithm

As early as 1763, the mathematician Reverend Thomas Bayes proposed the idea of Bayesian network algorithm [10]. Judea Pearl et al. constructed the first Bayesian network model based on graph theory and probability theory based on this idea in 1988. Subsequently, Mohammad et al. further studied the Bayesian algorithm and used the algorithm in the field of data mining applications, which received extensive attention in related fields [11]. The Naive Bayesian classification algorithm (Naive Bayesian, NB) is derived from the Bayesian network algorithm. It has the characteristics of simple structure and high classification accuracy. Although the algorithm is limited by the assumption of strong independence between attributes, it is in terms of classification ability. It is better than decision tree C4.5, SVM, KNN, and other algorithms [12, 13].

#### 2.4.1. Prior Probability and Posterior Probability

Assuming that events *M* and *N* are random events, and *P*(*M*) > 0, *P*(*N|M*) is the probability of event N occurring in a given *M* event, which is the posterior probability. Formula (3) can be used to express the relationship between *P*(*N|M*), *P*(*M*), and *P*(*M*∩*N*). Among them, *P*(*M*) is called the prior probability. Similarly, The relationship between the three *P*(*M|N*), *P*(*N*), *P*(*M*∩*N*) is as follows:

(3) $$\begin{array}{c} P\left(N|M\right)=\frac{P\left(M\cap N\right)}{P\left(M\right)}, \end{array}$$

(4) $$\begin{array}{c} P\left(M|N\right)=\frac{P\left(M\cap N\right)}{P\left(N\right)}. \end{array}$$

#### 2.4.2. Joint Probability

The joint probability means that two events happen at the same time. If *M* and *N* are two random events, then *P*(*M*∩*N*) can be used to represent the joint probability of *M* and *N*. The calculation formula is as follows:

(5) $$\begin{array}{c} P\left(M\cap N\right)=P\left(N|M\right)*P\left(M\right). \end{array}$$

Respectively, use *M*_1_, *M*_2_, *M*_3_,…, *M*_*i*_ to represent *i* random events, and then (5) can be transformed into the following equation:

(6) $$\begin{array}{c} P\left(M_{1},M_{2},M_{3},\ldots ,M_{i}\right)=P\left(M_{1}\right)*P\left(M_{2}|M_{1}\right)*\cdots *P\left(M_{i}|M_{1},M_{2},\ldots ,M_{n-1}\right). \end{array}$$

When *M* and *N* are independent events, there are

(7) $$\begin{array}{c} P\left(M\cap N\right)=P\left(N|M\right)*P\left(M\right)=P\left(N\right)*P\left(M\right). \end{array}$$

When *M*_1_, *M*_2_, *M*_3_,…, *M*_*i*_ are all independent of each other, then there is

(8) $$\begin{array}{c} P\left(M_{1},M_{2},M_{3},\ldots ,M_{i}\right)=P\left(M_{1}\right)*P\left(M_{2}\right)*P\left(M_{3}\right)*\cdots *P\left(M_{i}\right). \end{array}$$

The article "Application of Ultrasound Virtual Reality in the Diagnosis and Treatment of Cardiovascular Diseases" was published in 2021. Journal: J Healthc Eng.

#### 2.4.3. Full Probability

Let *N*_1_, *N*_2_, *N*_3_,…, *N*_*i*_ be the *i* partitions in the sample space *V*, where *P*(*N*_*j*_)〉0(*j*=1,2,3,…, *i*), Then, the total probability formula of event *M* is

(9) $$\begin{array}{c} P\left(M\right)=P\left(M|N_{1}\right)P\left(N_{1}\right)+\cdots +P\left(M|N_{i}\right)P\left(N_{i}\right)=\sum_{j=1}^{i}P\left(M|N_{j}\right)P\left(N_{j}\right). \end{array}$$

#### 2.4.4. Maximum Likelihood Probability

For a given data set *Y*, the classifier finds *C*_*j*_ that meets the largest possible hypothesis from category *C*, where *C*_*j*_ belongs to *C*, That is to say, this hypothesis is called the maximum posterior hypothesis, also called the maximum likelihood probability, denoted as *l*_max_, that is, according to the Bayesian formula,

(10) $$\begin{array}{c} l_{\max}=\underset{C_{j}\in C}{\arg\;\max}P\left(C_{j}|Y\right)=\underset{C_{j}\in C}{\arg\;\max}\frac{P\left(Y|C_{j}\right)P\left(C_{j}\right)}{P\left(Y\right)}. \end{array}$$

From the formula, *P*(*Y*) is a constant that has nothing to do with *C*_*j*_, so it can be simplified to

(11) $$\begin{array}{c} l_{\max}=\underset{C_{j}\in C}{\arg\;\max}P\left(C_{j}|Y\right)=\underset{C_{j}\in C}{\arg\;\max}P\left(Y|C_{j}\right)P\left(C_{j}\right). \end{array}$$

From formulas (3) and (4), we can get

(12) $$\begin{array}{c} P\left(M|N\right)*P\left(N\right)=P\left(N|M\right)*P\left(M\right). \end{array}$$

Transform formula (12) into

(13) $$\begin{array}{c} P\left(N|M\right)=\frac{P\left(M|N\right)*P\left(N\right)}{P\left(M\right)}. \end{array}$$

Substitute the total probability formula (9) into formula (13) to obtain the formula (14), which is called the Bayes formula.

(14) $$\begin{array}{c} P\left(N|M\right)=\frac{P\left(M|N\right)*P\left(N\right)}{P\left(M\right)}=\frac{P\left(M|N\right)*P\left(N\right)}{\sum_{j=1}^{i}P\left(M|N_{j}\right)*P\left(N_{j}\right)}. \end{array}$$

Assuming that the data set has *i* attributes, the conditional attribute value of the sample to be classified is *Y*, where *Y*={*a*_1_, *a*_2_,…, *a*_*i*_}, according to Bayes' theorem, obtains the following formula:

(15) $$\begin{array}{c} P\left(C_{j}|Y\right)=\frac{P\left(Y|C_{j}\right)}{P\left(Y\right)}P\left(C_{j}\right). \end{array}$$

Among them, *P*(*Y|C*_*j*_) is the conditional probability of feature vector *Y* in category *C*_*j*_, and *P*(*C*_*j*_) is the prior probability of category *C*_*j*_, According to the related knowledge of probability theory introduced above, the following formula is obtained:

(16) $$\begin{array}{c} P\left(Y\right)=\sum_{j=1}^{i}P\left(Y|C_{j}\right)P\left(C_{j}\right). \end{array}$$

Naive Bayes decision criterion: for any *j* ≠ *n*, there is *P*(*C*_*j*_*|Y*)〉*P*(*C*_*n*_*|Y*), and then the category of the attribute set *Y* is judged to be *C*_*j*_. Since *P*(*Y*) has nothing to do with *C*, the formula of the Naive Bayes classifier model is as follows:

(17) $$\begin{array}{c} C\left(Y\right)=\arg\;\max P\left(C_{j}\right)P\left(Y|C_{j}\right). \end{array}$$

Since the Naive Bayes classifier assumes that the attributes are independent of each other, there are

(18) $$\begin{array}{c} P\left(Y|C_{j}\right)=\prod_{k=1}^{i}P\left(Y_{k}|C_{j}\right). \end{array}$$

Therefore, the revised formula is

(19) $$\begin{array}{c} C\left(Y\right)=\arg\;\max P\left(C_{j}\right)\prod_{k=1}^{i}P\left(Y_{k}|C_{j}\right). \end{array}$$

The article "Application of Ultrasound Virtual Reality in the Diagnosis and Treatment of Cardiovascular Diseases" was published in 2021. Journal: J Healthc Eng.

### 2.5. Surgical Simulation System

Surgery simulation system is one of the examples of the combination of scientific computing visualization and virtual reality technology used in medicine [14, 15]. Surgical simulation system has a huge promotion effect on traditional clinical medicine. It benefits not only patients, but also doctors. The key to the surgical simulation system is its individualization, because each patient's anatomy is different. Compared with anatomical and surgical Atlas, changes in pathological factors can cause local conditions, which are individualities based on commonality. Surgery simulation system can reduce the risk of surgery and allow doctors to better control the success rate of surgery. From an educational point of view, young doctors use surgical experience and the role models of experts and researchers, which greatly saves the cost and time of training medical staff and further greatly reduces the risk of unskilled personnel performing surgery. Hospitals can improve the efficiency and quality of clinical surgical skills training and improve the uneven development of surgical skills in my country.

In terms of clinical application, even experienced professionals are at high risk in certain difficult situations. Preoperative surgical arrangements and surgical simulation procedures can completely reduce the incidence of surgical complications [16]. The biggest difference between surgical simulation systems and traditional imaging is not only in two-dimensional image analysis, but also in their accessibility and flexibility. In the surgical simulation system, the operator can arbitrarily control the position of the object, move and rotate arbitrarily, and perform various detailed and precise operations. This kind of operation requires a good coordination between hands and eyes [17]. For example, in a surgical simulation system, the resistance of the simulated equipment and absolute care can enhance the sense of surgery under the microscope and improve the microsurgery skills of young doctors. Wearing special glasses, you can observe 3D images and 3D senses and sights. The sense of environment that can create a personal experience makes people feel that the image is hovering on the screen [18]. The application of the surgical simulation system to the diagnosis of cardiovascular diseases can further show the complex three-dimensional spatial structure of the heart on the basis of echocardiography and can make three-dimensional measurement, defect closure simulation, and other measures to assist doctors in diagnosis and treatment, which will be an important development trend [19, 20].

The article "Application of Ultrasound Virtual Reality in the Diagnosis and Treatment of Cardiovascular Diseases" was published in 2021. Journal: J Healthc Eng.

## 3. Application Experiment of Ultrasound Virtual Reality Technology in the Diagnosis and Treatment of Cardiovascular Diseases

### 3.1. Main Content of the 3D Ultrasonic Virtual Measurement System

#### 3.1.1. Filtering of Ultrasound Image Data

Filtering is the preliminary step of segmentation. A suitable filter method can eliminate some interference and provide the necessary prerequisites for more accurate segmentation. The filtering method in this paper adopts the multiscale heterogeneous anisotropic diffusion method combined with median filtering.

#### 3.1.2. Segmentation of Ultrasound Image Data

Segmentation is the key content of data processing. The segmentation in this study is to divide the image into two parts of the myocardium and cardiac cavity, in preparation for achieving a better three-dimensional visualization effect. The segmentation method uses the level set method combined with fuzzy mean clustering without reinitialization. In the segmentation method, in order to improve the evolution efficiency of the level set and reduce the number of iterations, the initial function of the level set is determined by the membership degree. In order to reduce the occurrence of segmentation errors, a fuzzy membership function is added to the level set area functional. The stop function of the control.

The article "Application of Ultrasound Virtual Reality in the Diagnosis and Treatment of Cardiovascular Diseases" was published in 2021. Journal: J Healthc Eng.

#### 3.1.3. Three-Dimensional Measurement System in Virtual Reality

The realization of the 3D heart measurement system is based on the 3D rendering and interaction system. The main content of the three-dimensional measurement system is the acquisition of the coordinates of the point in the virtual reality, and the measurement of distance and area in the three-dimensional environment. Finally, the results of 3D virtual measurement are given. The basic process is: image data acquisition and reconstruction ⟶ image data filtering and segmentation ⟶ 3D visualization and virtual reality ⟶ 3D virtual measurement system [21, 22].

### 3.2. Data Collection

The data used are provided by two acquisition methods: transthoracic multi-planar probe (TTO) sampling method and full volume (Full Volume) sampling method. HP SONOS 5500 and HP SONOS 7500 color Doppler echocardiography were used for sampling.

#### 3.2.1. TTO Sampling Method

The sampling diagram of the TTO sampling function is shown in the figure below. The sampling method of the detector is shown in Figure 1. The detector rotates 360° along its central axis to perform a full-scale scan. The imaging will be synchronized with the cardiac cycle to capture a series of two-dimensional cross-sectional images. The ultrasound scanner can choose to scan each rotating part at 1°2°3° and obtain 180/90/60 original ultrasound images of the heart, including the two-dimensional image information of the entire heart. The size of the collected image is 240 pixels × 128 pixels, with 256 levels of gray.

#### 3.2.2. Full Volume Sampling Method

Full Volume is a sample of the entire volume of the entire heart, also known as the representation of a wide-angle pyramid. In other words, a set of four real-time 3D melon petals (0°∼15°, 15°∼30°, 30°∼45°, 45°∼60°) are collected in sequence and integrated into the pyramid to integrate the entire heart. The volume data set: once digitized, it will be saved on the 3D hard drive in DICOM format. Therefore, the data in DICOM format will be sorted according to the actual data location and include cardiac cycle movements.  Figure 2 shows a schematic diagram of the full volume acquisition.

#### 3.2.3. Comparison of Two Sampling Methods

The range of images collected by these two capture methods is wide, and the entire image of the detection target can be displayed, because these images are realistic, the proximity to each structure is clearly visible, and there are almost no defects in the heart wall. It is very helpful for observing stroke volume, myocardial infarction, myocardial weight, and heart wall dynamics and for myocardial perfusion imaging.

The Full Volume acquisition method takes about 5 to 7 seconds for one sampling. If the patient can hold their breath without moving, the offset between the four narrow-angle images to be taken will be very small. The disadvantage is that the image consists of four real-time 3D images with four consecutive cardiac cycles. In the case of dislocation or arrhythmia, it may cause image distortion.

The article "Application of Ultrasound Virtual Reality in the Diagnosis and Treatment of Cardiovascular Diseases" was published in 2021. Journal: J Healthc Eng.

However, the TTO collection method requires more than 3 minutes for one sampling, which requires relatively high requirements for patients. However, due to the higher resolution of the collection, the accuracy of the data is greater.

### 3.3. 3D Data Reconstruction

For the data collected in the above two ways, different methods are used to reconstruct the data.

#### 3.3.1. TTO Sampling Method

For the TTO acquisition method, since the sampling method of the ultrasonic probe is a full-scale sector scan, the secondary transformation method of sector scan is used to reconstruct and combine the data, and finally the displayed image is obtained. The schematic diagram of this method is shown in Figure 3.

Figure 3(a) shows the sampling level of the ultrasound scan, the ultrasound detector sends *N* sampling lines for on-site scanning, and Figure 3(b) shows the image storage level. The image memory is a large-capacity storage body installed on a matrix that stores the echo image data sampled on the sampling surface of the ultrasound scanner, reads it according to a specific time sequence, and uses it for image processing after processing. At the memory level, the modulus *R* and the argument *α*, sampled in polar coordinates, correspond to the row and column addresses in the memory. First, the points in the sampling plane, that is, the aforementioned linear *N*-scan data, are stored in the memory, and then the Cartesian coordinates of the points in the area displayed in the display plane are converted to the next level. The data in the memory above the memory level undergoes two-line interpolation to obtain coordinate values. With the correct spatial transformation, a series of 2D images can be recreated in a three-dimensional Cartesian coordinate system, where the pixels are evenly distributed. Use linear interpolation to obtain the gray point value of the replacement pixel. The size of the reconstructed 3D volume data is 240 × 240 × 128.

#### 3.3.2. Full-Volume Sampling Method

For the Full-Volume acquisition method, the collected data is stored in a file in DICOM format. DICOM file is a special format with the suffix.dcm, used to store medical images. This format is widely used in hospital CT, MRI, and PACS systems, but image readers usually do not support this image format. The DICOM standard uses the information object definition IOD model to abstractly describe these objects. Each object contains many attributes, and each attribute is represented by a data element. A data element generally consists of a tag (tag), a value description (VR), a value length (VL), and a value field (value field). Each data element has a unique label, and multiple elements are arranged from small to large according to the label, which is called a data set.

The article "Application of Ultrasound Virtual Reality in the Diagnosis and Treatment of Cardiovascular Diseases" was published in 2021. Journal: J Healthc Eng.

In the Full Volume acquisition method, the collected data will be interpolated and adjusted according to the standard and stored in the DICOM format data in the order of height, width, depth, and time. Therefore, the data can be separated in time without the need for a separate reconstruction process. The size of the 3D volume data obtained depends on the data collection state at the time of collection.

### 3.4. Filtering and Segmentation of Three-Dimensional Heart Images

Multiscale heterogeneous anisotropic diffusion method is used to process the data. This method uses the median anisotropic diffusion algorithm to deconstruct the ultrasonic speckle noise. There are two differences between this method and the traditional anisotropic diffusion technology: (1) there are two resolutions. Low-resolution images convert speckle noise into quasi-impulse noise, making speckle noise easier to remove. (2) A median term is applied to the anisotropic diffusion equation, making it more suitable for removing impulsive noise.

The main body of segmentation is an improved level set method without reinitialization. In order to improve the evolution efficiency of the level set and reduce the number of iterations, the initial function of the level set is determined by the degree of membership; and in order to reduce the occurrence of segmentation errors, the area of the level set is generalized. A stop function S controlled by the fuzzy membership function *y* is added to the function. The overall frame of the segmentation is shown in Figure 4:

### 3.5. 3D Visualization and Virtual Reality Environment

The Visualization Toolkit (VTK) is a supporting environment for the construction and operation of visualization applications. It is developed on the basis of the three-dimensional function library OpenGL, using object-oriented design methods. It shields the details that are often encountered in the visual development process and encapsulates some commonly used algorithms. Then, use the improved Marching Cubes algorithm to implement an interactive virtual reality environment for the built three-dimensional data set.

In order to reflect the effect of virtual reality, it is necessary to provide users with interactive operation tools—mouse interaction and keyboard interaction. Through these two methods, the effect of the basic virtual endoscope is realized. For example, place the view in the heart, roam the observation angle, change the observation distance, adjust the observation angle, and dynamically design and display the web structure in front of the observation angle in real time. This method can effectively see whether there are lesions inside the organ, which is convenient for doctor observation and diagnosis.

The article "Application of Ultrasound Virtual Reality in the Diagnosis and Treatment of Cardiovascular Diseases" was published in 2021. Journal: J Healthc Eng.

### 3.6. Three-Dimensional Heart Measurement

The basic steps of using a computer to measure three-dimensional objects are as follows: (1) data acquisition, (2) data preprocessing, (3) three-dimensional display and observation, and (4) three-dimensional interactive measurement.

## 4. Application Analysis of Ultrasound Virtual Reality Technology in the Diagnosis and Treatment of Cardiovascular Diseases

### 4.1. Analysis of Filtering and Segmentation of Three-Dimensional Heart Images

In order to show the two-dimensional filtering effect of several data, the middle section of the two-dimensional data is extracted. It can be seen that speckle noise has been effectively suppressed, while important information (such as the strength and edges of the anatomical structure) is basically maintained. It is difficult to give a quantitative evaluation of the filtering effect. Because it is impossible to know what the ideal image looks like, it is impossible to obtain a quantitative result that the filtered image is closer to the ideal image compared to the prefiltered image. However, the evaluation of the histogram of the uniform area of the image can yield a more convincing metric. Generally, if the filtered image is “better” than the prefiltered image, then (in a relatively uniform area) the image histogram must be narrower; that is, the noise will be smaller. The filtered image can remove a lot of noise while keeping the basic gray information of the original image unchanged and achieve a better filtering effect.

### 4.2. Three-Dimensional Heart Measurement Analysis

The study object was isolated pig hearts, and 10 isolated congenital heart disease models with atrial septal defect (ASD) were established. The image acquisition instrument is a SONOS 5500 echocardiograph. The ultrasound detector rotates once every 1° to perform a sector scan to collect 180 original cardiac ultrasound slices and obtain a 3D data set, and this 3D data set contains the 2D information of the entire heart. Perform ultrasound 3D virtual reality imaging on the isolated atrial septal defect model, check the angle of view, and observe the 3D atrial septal defect from the horizontal axis and vertical axis of the left and right atrium of the septal defect, and the entire range of the septal defect.  Figure 5 is a two-dimensional slice of ventricular tissue.

The article "Application of Ultrasound Virtual Reality in the Diagnosis and Treatment of Cardiovascular Diseases" was published in 2021. Journal: J Healthc Eng.

Regarding the statistics on the results of 10 cases of ASD model measurement, it can be found that the data of real measurement and virtual measurement are basically close (the unit of length is millimeters, and the unit of area is square millimeters). The real measurement and virtual measurement results of the left atrium are shown in Table 1 and Figure 6.

The real measurement and virtual measurement results of the right atrium are shown in Table 2 and Figure 7.

The measurement results are statistically analyzed, and the results are shown in Tables 3 and 4. *L* value less than 0.05 indicates that the statistics are meaningful: *R* value generally greater than 0.9 indicates that the virtual measurement results are highly correlated with the real measurement results. This proves that the virtual measurement system can achieve relatively accurate measurement of clinical data, and the virtual measurement results can be used as reference data for doctors' diagnosis.  Figure 8 shows the statistics of the real data and virtual measurement results of the left and right atria.

## 5. Conclusions

The application of three-dimensional visualization and virtual reality technology to the research of cardiovascular diseases can simulate the structure and condition of the diseased heart in a computer, which is convenient for doctors to make further diagnosis and treatment. Surgery simulation system can not only help doctors make qualitative judgments, but also make quantitative measurements. Although the imaging quality of ultrasound images is not as good as that of CT and MRI, the advantages of noninvasiveness and economy have made it one of the most commonly used medical imaging methods. I believe that through the development of ultrasound imaging systems and computer technology in the future, the development of this field will become deeper and deeper, and the application will become more and more extensive. The disadvantage of this article is that the virtual measurement data of the three-dimensional heart is too few, and the design of the entire surgical simulation system is not perfect.

## Figures and Tables

**Figure 1:** The position and sampling plane of the rotating probe in the TTO sampling method.

**Figure 2:** Full volume sampling.

**Figure 3:** Schematic diagram of ultrasound image acquisition. (a) Memory plane. (b) Image memory plane. (c) Display plane.

**Figure 4:** Split the overall framework.

**Figure 5:** Two-dimensional slice of the ventricle (this picture is borrowed from Baidu encyclopedia).

The article "Application of Ultrasound Virtual Reality in the Diagnosis and Treatment of Cardiovascular Diseases" was published in 2021. Journal: J Healthc Eng.

**Figure 6:** The real and virtual measurement results of the left atrium.

**Figure 7:** The real and virtual measurement results of the right atrium.

**Figure 8:** Statistics of real data and virtual measurement results of the left and right atria.

**Table 1:** Real and virtual measurement results of the left atrium.

Measurement content	Number	Minimum value	Max	Mean	Standard deviation
ASD long	10	7.8	13.8	11.180	2.2566
ASD long (virtual)	10	7.9	14.6	11.460	2.4197
ASD short	10	3.8	12.3	7.750	2.4985
ASD short (virtual)	10	3.5	10.9	7.120	2.0263
ASD area	10	20.3	137.4	72.310	35.2640
ASD area (virtual)	10	20.9	132.5	68.870	32.5892

**Table 2:** Real and virtual measurement results of the right atrium.

Measurement content	Number	Minimum value	Max	Mean	Standard deviation
ASD long	10	6.3	12.5	11.020	2.1258
ASD long (virtual)	10	6.2	12.1	11.240	2.2897
ASD short	10	4.0	11.8	7.680	2.3524
ASD short (virtual)	10	4.2	11.2	7.090	2.0118
ASD area	10	21.8	141.3	72.260	34.2386
ASD area (virtual)	10	20.6	135.8	68.840	32.7873

**Table 3:** The relationship between real data and virtual measurement results of the left atrium.

Measurement content	*R*	*L*
Measure the ASD long diameter in the left atrium	0.956	0.000
ASD short diameter measured in the left atrium	0.928	0.000
ASD area measured in the left atrium	0.975	0.000

**Table 4:** The relationship between the real data of the right atrium and the virtual measurement results.

Measurement content	*R*	*L*
Measure the ASD long diameter in the right atrium	0.927	0.000
ASD short diameter measured in the right atrium	0.949	0.000
ASD area measured in the right atrium	0.968	0.000

## Data Availability

Data sharing is not applicable to this article, as no datasets were generated or analyzed during the current study.
